The article "Maternal Smoking and the Risk of Placenta Accreta Spectrum: A Systematic Review and Meta-Analysis" was published in 2022. Journal: Biomed Res Int.

# Maternal Smoking and the Risk of Placenta Accreta Spectrum: A Systematic Review and Meta-Analysis

**DOI:** 10.1155/2022/2399888

**Published:** 2022-07-11

**Authors:** Ensiyeh Jenabi, Amir Mohammad Salehi, Seyedeh Zahra Masoumi, Azam Maleki

**Affiliations:** ^1^Autism Spectrum Disorders Research Center, Hamadan University of Medical Sciences, Hamadan, Iran; ^2^School of Medicine, Hamadan University of Medical Sciences, Hamadan, Iran; ^3^Mother and Child Care Research Center, School of Nursing and Midwifery, Hamadan University of Medical Sciences, Hamadan, Iran; ^4^Social Determinants of Health Research Center, Zanjan University of Medical Sciences, Zanjan, Iran

## Abstract

**Background:**

This is the first meta-analysis that assessed the association between maternal smoking and the risk of placenta accreta spectrum (PAS), so this study was aimed at investigating the association between maternal smoking and PAS based on observational studies. PAS is defined as a severe obstetric complication due to the abnormal invasion of the chorionic villi into the myometrium and uterine serosa.

**Methods:**

We searched electronic bibliographic databases including PubMed, Web of Science, Scopus, Science Direct, and Google Scholar until January 2022. The results were reported using a random effect model. The chi-square test and the *I*^2^ statistic were used to assess heterogeneity. Egger's and Begg's tests were used to examine the probability of publication bias. All statistical analyses were performed at a significance level of 0.05 using Stata software, version 11.

**Results:**

Based on the random effect model, the estimated OR of the risk of PAS associated with smoking was 1.21 (95% CI: 1.02, 1.41; *I*^2^ = 4.7%). Subgroup analysis was conducted based on study design, and the result showed that the association between smoking and PAS among cohort studies was significant 1.35 (95% CI: 1.15, 1.55; *I*^2^ = 0.0%).

**Conclusion:**

Our results suggested that maternal smoking is a risk factor for the PAS. There was no heterogeneity among studies that reported an association between smoking and the PAS. The Newcastle-Ottawa Scale (NOS) was used to measure study quality.

## 1. Introduction

Placenta accreta spectrum (PAS), formerly known as adherent placenta, is a term used to describe the abnormal attachment of placental trophoblasts to the uterine myometrium and includes placenta accreta (placenta attachment to myometrium without decidua intervention), increta placenta (trophoblast invasion to myometrium), and percreta placenta (invasion through the myometrium is serous and into the surrounding structures) [1].

The importance of this disease is due to the increase in maternal and fetal mortality. Fetal outcomes are mainly due to iatrogenic prematurity, while maternal outcomes are mainly due to increased risk of postpartum hemorrhage and surgical complications. The average blood loss is 3000-5000 ml, and up to 90% of patients need a blood transfusion [2]. Complications of surgery include hysterectomy and injury to the ureter, bladder, and intestines, which leads to more intensive care admissions and longer hospital stays, as well as posttraumatic stress disorder (PTSD) and more psychological consequences [3].

Diagnosis of the PAS is based on two main clinical and pathological criteria. After delivery, the placenta usually separates spontaneously, and any difficulty in separating the placenta or the need for placental abruption is considered a clinical criterion for the PAS. Another clinical criterion is uncontrollable bleeding from the placenta after delivery or cesarean section [4]. Prenatal diagnosis of PAS is usually made by ultrasound [5, 6].

In the umbrella review of Jenabi et al., multiple gestation and in vitro fertilization (IVF) were identified as definitive risk factors [7]; also, in other studies, uterine surgery, placenta previa, and advanced maternal age have been introduced as risk factors [8–10]. Recently, several studies have warned about the dangers of smoking, diet, and chronic condition and their association with PAS.

The role of smoking in some diseases is also known such as esophageal cancer [11] and hypertension [12], placenta previa [13], and placenta abruption [14]; however, no meta-analysis study has quantitatively assessed the association between maternal smoking and the risk of PAS, so this study was aimed at investigating the association between maternal smoking and PAS based on observational studies. Herein, we performed the first meta-analysis to identify role association between maternal smoking and PAS.

## 2. Methods

The checklist of the Preferred Reporting Items for Systematic Reviews and Meta-Analyses (PRISMA) was used for performing the present meta-analysis. Investigating the association between maternal smoking and risk of PAS was performed regarding to the following PICO framework:

- Population: pregnant women
- Intervention: smoking before and during pregnancy
- Comparison: without smoking before and during pregnancy
- Outcome: risk of placenta accreta spectrum

Observational studies (case-control and cohort) reporting the association between smoking and the risk of PAS were reviewed, irrespective of language, maternal age, race, country, date, and place of publication.

The search strategy was based on combining a set of keywords (“placenta accreta” or “placenta increta” or “placenta percreta” or “placenta accreta spectrum” or “morbidly adherent placenta” or “abnormally invasive placenta”) and (“Smoking” or “cigarette” or “tobacco” or “cigar”). We searched electronic bibliographic databases including PubMed, Web of Science, Scopus, Science Direct, and Google Scholar until January 2022. To find additional references, we screened the reference lists of the included studies. In addition, we contacted authors of the studies to earn eligible studies, and conference databases were searched.

Two authors independently reviewed the articles to ensure that they met the meta-analysis inclusion criteria. Any disagreements among the authors were resolved by discussion. The two authors extracted information from the included articles. The information was the first author's name (year), country, study design, age (year), sample size, and the effect measure and its 95% confidence interval (CI). The Newcastle-Ottawa Scale (NOS) was used to measure study quality [15]. A study had a maximum of 9 NOS stars: 4 stars for quality of selection, 2 stars for comparability, and 3 stars for quality of exposures. Studies with NOS scores of 7 and higher were categorized as high quality, while studies with NOS scores of 6 and less were categorized as low quality.

The chi-square test and the *I*^2^ statistic were used to assess heterogeneity [16]. Egger's [17] and Begg's [18] tests were used to examine the probability of publication bias.

Odds ratio (OR), with their associated 95% CIs, were applied to present the measures of association between maternal smoking and PAS. We used the adjusted forms of the ORs, controlling for at least one of the potential confounding factors. The results were reported using a random effect model. We conduct a subgroup analysis based on study design and crude/adjust form. All statistical analyses were performed at a significance level of 0.05 using Stata software, version 11 (StataCorp, College Station, Texas, USA).

## 3. Results

### 3.1. Description of Studies

Until 30 January 2022, 321 studies were included in the present meta-analysis. Of these, 176 were excluded due to duplication and 145 studies remained for assessing title and abstract. Then, 128 studies were excluded after reading titles and abstracts. In total, 17 studies were remained for reading the full papers. Three full papers were not considered to be eligible (four studies were reviewed and three studies had no inclusion criteria). In the end, 14 studies were included in the current meta-analysis (Figure 1). We identified ten studies with cohort [3, 19–27] and four studies [28–31] with case-control designs. The participants in this study were 3,892,832. All studies were in English (Table 1).

### 3.2. Effects of Exposure

Figure 2 presented the association between smoking and the PAS. Based on the random effect model, the estimated OR of the risk of PAS associated with smoking was 1.21 (95% CI: 1.02, 1.41; *I*^2^ = 4.7%). The finding of Farquhar's study [29] was reported among primiparous and multiparous, separately.

### 3.3. Publication Bias

Publication bias was carried out using Begg's and Egger's tests. The *p* values for Begg's and Egger's regression were 0.656 and 0.439, respectively. Evidence of publication bias was not seen among studies showing the association between smoking and PAS in Figure 3.

### 3.4. Subgroup Analysis

Subgroup analysis was conducted based on study design, and the result showed that the association between smoking and PAS among cohort studies was significant 1.35 (95% CI: 1.15, 1.55; *I*^2^ = 0.0%), but this association among case-control studies was not significant 0.83 (95% CI: 0.47, 1.19; *I*^2^ = 0.0%). In addition, there was no significant association between smoking and PAS based on crude/adjust form (Table 2).

### 3.5. Quality of the Studies

According to the NOS, 12 studies were high quality and 2 studies were low quality (Table 1).

## 4. Discussion

To the best of our knowledge, this is the first meta-analysis that reports the association between maternal smoking and the risk of PAS based on observational studies. Our findings reported that maternal smoking is a risk factor for the PAS. There was no heterogeneity among studies that reported an association between smoking and the PAS.

A meta-analysis was conducted in 2020 by Iacovelli et al. [32]. They reported that current smoking is not a risk factor for abnormally invasive placenta (OR = 1.13; 95% CI: 0.88, 1.47). They searched PubMed, Embase, and CINAHL databases with the design of case-control, case reports, and case series. However, they did not include all observational studies in the meta-analysis, and this can lead to bias among the results.

The rate of placenta accreta was reported from 0.001% to 0.9% of deliveries [33]. The incidence of placenta accreta has increased 10-fold in the past 50 years that probably resulted from the elevated cesarean section rate [34]. Advanced maternal age, uterine anomalies, and previous uterine scar appear to work synergistically to increase the risk of placenta accreta [35].

The characteristics and consequences of the patient are different in the subgroups of the accreta placenta spectrum, and women with the placenta increta and percreta have a high risk of morbidity and surgical mortality [22].

Elevated first-trimester serum placental growth factor (PIGF) was significantly associated with placenta accreta, indicating the potential role of PIGF in identifying high-risk pregnancies for placenta accreta [19].

Several studies have shown that smoking causes hypercoagulability and increased risk of thrombosis, and during pregnancy, due to physiological adaptation, the hemostatic system presents as a relatively hypercoagulable state with decreased anticoagulation function; however, studies in women with PAS have shown that they have hypocoagulability and hyperfibrinolysis [36]; therefore, the mechanism of the association between smoking and the PAS is unknown. However, the systemic inflammation induced by air pollution affects female genital tract damage, including damage to the endometrial and myometrium epithelium, and leads to poor decidualization [37, 38]. Another study showed that exposure to an air pollutant (PM_2.5_) was associated with placenta inflammation [39]. Therefore, it seems that pollutant-induced inflammation during pregnancy could also cause inflammation in the endometrium, leading to the PAS [40].

According to Tsuji et al., cadmium and lead levels in pregnant women with PAS were higher than normal pregnancies, and it is possible that increased cadmium levels play a role in the pathogenesis of PAS [20]. Smoking can also increase cadmium levels in the blood [41]. However, further studies are needed to substantiate this hypothesis because cadmium and lead levels were also higher in women with PAS without a history of smoking than in women with normal pregnancies [20].

### 4.1. Limitations

This study has some limitations. In our meta-analysis, diagnosis of PAS was most by clinicians, and pathology reports were not obtained from all cases. Therefore, most of the PAS cases in this study were clinically diagnosed. In addition, some of the included studies in our meta-analysis adjusted for confounding variables. This was another limitation of this study. Also, all studies did not investigate the effect of smoking on the PAS in trimesters of pregnancy, separately. Therefore, we did not conduct a subgroup analysis based on time smoke use during pregnancy.

### 4.2. Strength points

One of the strengths of this study is the homogeneity of the studies included in the meta-analysis and their high quality; also, the present meta-analysis with 3,892,832 participants reported that maternal smoking is a risk factor for the PAS.

## 5. Conclusion

PAS is becoming increasingly common and is associated with significant morbidity and mortality. Knowledge of risk factors can help prevent and diagnose early. Our results suggested that maternal smoking is a risk factor for the PAS; also, there was no heterogeneity among studies that reported an association between smoking and the PAS.

## Figures and Tables

**Figure 1:** Flow of diagram of the systematic process.

**Figure 2:** Forest plot of the smoking and placenta accreta spectrum.

**Figure 3:** Funnel plot of the smoking and placenta accreta spectrum.

**Table 1:** Characteristics of the studies in the meta-analysis.

1^st^ aut, year	Design	Sample	Diagnose method	Maternal age (year)	Estimate	Adjustment	Quality
Usta, 2005 [28]	Case-control	347	By maternal–fetal medicine physicians	31	Odds ratio	Adjust	High
Matsuzaki, 2021 [22]	Cohort	2727477	ICD-10 codes	Not reported	Odds ratio	Adjust	High
Svanvik, 2021 [21]	Cohort	9376	Attending obstetrician and clinical diagnosis	Not reported	Odds ratio	Crude	High
Kyozuka, 2019 [3]	Cohort	90554	Histological examination or the clinical presentation	31.8	Odds ratio	Adjust	High
Wang, 2020 [19]	Cohort	177	Histological	30.22	Odds ratio	Crude	High
Bowman, 2014 [25]	Cohort	2749	Pathology or clinical findings	30.85	Odds ratio	Adjust	High
Tsuji, 2019 [20]	Cohort	16019	Medical record	32.7	Odds ratio	Crude	High
Eshkoli, 2013 [24]	Cohort	34869	Clinical	Not reported	Odds ratio	Crude	High
Farquhar, 2017 [29]	Case-control	865	Imaging or by pathological	Not reported	Odds ratio	Adjust	High
Jauniaux, 2019 [23]	Cohort	292	By physicians and ultrasound	34.30	Odds ratio	Crude	High
Upson, 2013 [26]	Cohort	403602	ICD-10	Not reported	Odds ratio	Crude	Low
Klar, 2013 [30]	Case-control	483	ICD	34.47	Odds ratio	Crude	Low
Fitzpatrick, 2012 [31]	Case-control	390	Histological	Not reported	Odds ratio	Crude	High
Ueno, 2014 [27]	Cohort	65	Pathological	Not reported	Odds ratio	Crude	High

**Table 2:** Results of subgroup analysis of the maternal smoking and placenta accreta spectrum based on study design and adjust/crude form for control of the counfounding variables.

Subgroups	No. of studies	OR (95% CI)	*I* ^2^
Study design			
Case-control	4	0.83 (0.47, 1.19)	0.0%
Cohort	10	1.35 (1.15, 1.55)	0.0%
Adjust/crude form			
Adjust analysis	6	1.11 (0.74, 1.49)	32.1%
Crude analysis	8	1.29 (1.0, 1.58)	0.0%

## Data Availability

Access to data is possible with permission from the responsible author.

## Abbreviations

PAS: Placenta accreta spectrum
NOS: Newcastle-Ottawa Scale
OR: Odds ratio
CI: Confidence interval
PRISMA: Preferred Reporting Items for Systematic Reviews and Meta-Analyses
PIGF: Placental growth factor.
